# A Novel Image Encryption Technique Based on Cyclic Codes over Galois Field

**DOI:** 10.1155/2022/1912603

**Published:** 2022-02-08

**Authors:** Muhammad Asif, Joshua Kiddy K. Asamoah, Mohammad Mazyad Hazzazi, Adel R. Alharbi, Muhammad Usman Ashraf, Ahmed M. Alghamdi

**Affiliations:** ^1^Department of Mathematics, University of Management and Technology, Sialkot Campus, Sialkot, Pakistan; ^2^Department of Mathematics, Kwame Nkrumah University of Science and Technology, Kumasi, Ghana; ^3^Department of Mathematics, College of Science, King Khalid University, Abha, Saudi Arabia; ^4^College of Computing and Information Technology, University of Tabuk, Tabuk 71491, Saudi Arabia; ^5^Department of Computer Science, GC Women University, Sialkot, Pakistan; ^6^Department of Software Engineering, College of Computer Science and Engineering, University of Jeddah, Jeddah, Saudi Arabia

## Abstract

In the modern world, the security of the digital image is vital due to the frequent communication of digital products over the open network. Accelerated advancement of digital data exchange, the importance of information security in the transmission of data, and its storage has emerged. Multiple uses of the images in the security agencies and the industries and the security of the confidential image data from unauthorized access are emergent and vital. In this paper, Bose Chaudhary Hocquenghem (BCH) codes over the Galois field are used for image encryption. The BCH codes over the Galois field construct MDS (maximum distance separable) matrices and secret keys for image encryption techniques. The encrypted image is calculated, by contrast, correlation, energy, homogeneity, and entropy. Histogram analysis of the encrypted image is also assured in this paper. The proposed image encryption scheme's security analysis results are improved compared to the original AES algorithm. Further, security agencies can utilize this work for their confidential image data.

## 1. Introduction

Nowadays, cryptography plays a primary role in information security and embedded system design. The use of mobile communication and the Internet rapidly increases and occupies wide-ranging areas in daily life. There is an increase in the number of users and unauthorized users who try to fetch data illegally, causing data security issues. To solve this problem, encrypted data is generated, unreadable for unauthorized users. Cryptography is the science of information security which secures the data while it is stored or transmitted. Claude Shannon [1] describes the two basic properties, diffusion and confusion for the design of block ciphers in a communication theory of secrecy systems. Substitution boxes are the block ciphers' only nonlinear component that confuses the ciphertext. Many researchers have created highly nonlinear and influential S-boxes to provide secure communication. The diffusion layer has been neglected in cryptographic research, juxtaposed to confusion layers for a long time. The replacement of the permutation layer of substitution-permutation networks (SPNs) by a diffusion layer enhances the avalanche property of the block cipher. It makes the cipher's resistance to linear and differential cryptanalysis explained by Heys and Tavare in [2–4]. Thus, MDS (maximum distance separable) matrices provide diffusion in cryptographic algorithms and are the main component in the architecture of block ciphers to make resistance against the linear and differential cryptanalysis. The keystream generator is added to the AES algorithm to improve encryption performance [5]. The modified AES algorithm is explained in [6]. The image and video encryption based on chaos with security analyses are presented in [7]. The existing image encryption techniques are reviewed in [8]. The article explains the simulation of image encryption using the AES algorithm [9]. Using Gaussian Distribution Cryptographic Substitution Box is designed in [10]. The present age ciphers SHARK [11], Advanced Encryption Standard (AES) [12], and Twofish [13,1 4] have a diffusion layer that depends on the mix column operation step. The least weight maximum distance separable (MDS) matrices constructed by comprehensive search from the companion matrices are given in [11]. Zhang et al. [15] presented chaotic research encryption, combining the image and DES encryption algorithm. Logistic chaos sequencer is used in the new encryption scheme to create the pseudorandom sequence and then makes double-time encryption with improvements in DES. Their results show high security and encryption speed and high starting value sensitivity. Shah et al. [16] propose a criterion to examine the prevalent S-boxes and study their strength and weaknesses to define their correctness in image encryption applications. The bases of the AES key expansion image encryption scheme are explained in [17]. Error-correcting codes, particularly BCH codes, are helpful to reduce the rate of decryption failure [18]. Walter et al. [18] analyze the decoding algorithm of the BCH code and design a constant-time version of the BCH decoding algorithm. Asif et al. [19] constructed BCH codes with a computational approach and applied those codes in data security. Different image encryption techniques are utilized by various authors [20–24].

The modified AES algorithm for image and text encryption based on bit permutation instead of mixed column operation is presented in [25]. But we used BCH codes to construct MDS matrices and private keys to secure image data. The proposed criteria use correlation analysis, entropy analysis, homogeneity analysis, contrast analysis, energy analysis, and histogram analysis. This paper presents a new symmetric algorithm based on BCH codes over the Galois field. MDS matrices and secrete keys of the proposed algorithm are derived from the generator polynomials of the respecting BCH codes over the Galois field. We furnished a novel technique for constructing the building components of the block cipher. The rest of the paper is organized as follows: some basic concepts of coding theory and cryptography are presented in Section 2.  Section 3 contains the proposed algorithm and its components with an example.  Section 4 has statistical analyses of the encrypted image by the proposed algorithm. Conclusion and future application are discussed in Section 5.

## 2. Preliminaries

### 2.1. Cyclic Codes

The linear mapping *ρ* : ℱ^*n*^⟶ℱ^*n*^ is defined by

(1) $$\begin{array}{c} \rho \left(b_{1},b_{2},b_{3},\ldots ,b_{n}\right)=\left(b_{n},b_{1},b_{2},b_{3},\ldots ,b_{n-1}\right). \end{array}$$

It is called a cyclic shift. A linear code *C* ⊂ ℱ^*n*^ is called cyclic code if

(2) $$\begin{array}{c} \rho \left(b\right)\in C,\;\forall b\in C. \end{array}$$

### 2.2. Irreducible Polynomial

A polynomial is called irreducible if it cannot be written as the product of two polynomials. For example, *P*(*x*)=*x*^3^+*x*+1 is an irreducible polynomial of degree 3 over *ℤ*_2_.

### 2.3. Primitive Polynomial

An irreducible polynomial *P*(*x*) is primitive polynomial if *α* is a primitive root of *P*(*x*), that is,

(3) $$\begin{array}{c} P\left(\alpha \right)=0,\\ \alpha^{p^{m}-1}=1, \end{array}$$

where *p* is prime and *m* is the degree of the irreducible polynomial. For example, *P*(*x*)=*x*^4^+*x*+1 is a primitive, irreducible polynomial over *ℤ*_2_.

### 2.4. Theorem [26]

Let *αϵ*ℱ_*q*^*m*^_. Then, *α*, *α*^*q*^, *α*^*q*^2^^, *α*^*q*^3^^,… have the same minimal polynomial over ℱ_*q*_.

### 2.5. BCH Code

BCH codes are cyclic linear codes. Let *c*, *d*, *q*, *n* be positive integers such that 2 ≤ *d* ≤ *n*, *q* is a power of some prime number, and (*n*, *q*)=1. Let *m* be the least positive integer such that

(4) $$\begin{array}{c} q^{m}\equiv 1\left(\mathrm{mod}n\right). \end{array}$$

Thus, *n|q*^*m*^ − 1. Let *α* be a primitive nth root of unity in *Ϝ*_*q*^*m*^_. Let *m*_*i*_(*x*) ∈ *Ϝ*_*q*_[*x*] denote the minimal polynomial of *α*^*i*^. Let *g*(*x*) be the product of distinct minimal polynomials among *m*_*i*_(*x*), *i*=*c*, *c*+1,…, *c*+*d* − 2, that is,

(5) $$\begin{array}{c} g\left(x\right)=l\cdot c\cdot m\left\{m_{i}\left(x\right)|i=c,c+1,\ldots ,c+d-2\right\}. \end{array}$$

Since *m*_*i*_(*x*) divides *y*^*n*^ − 1 for each *i*, it follows that *g*(*x*) divides *x*^*n*^ − 1. Let *C* be a cyclic code with generator polynomial *g*(*x*) in the ring *Ϝ*_*q*_[*x*]_*n*_. Then, *C* is called a BCH code of length *n* over *Ϝ*_*q*_ with designed distance *d*.

Nowadays, BCH codes have many applications; BCH codes are used in satellite communication, hard disc, compact disc, storage systems, and data security.

### 2.6. Theorem [26]

Let *C* be BCH code of length *n* over ℱ_*q*_ with designed distance *d*. Then

(6) $$\begin{array}{c} C=\left\{c\left(x\right)\in {ℱ}_{q}{\left[x\right]}_{n}:c\left(\alpha^{j}\right)=0,\;\forall j=c,c+1,c+2,\ldots ,c+d-2\right\}. \end{array}$$

### 2.7. Theorem [26]

Let *C* be a BCH code of designed distance *d*. Then,

(7) $$\begin{array}{c} d\left(c\right)\geq d, \end{array}$$

where *d*(*c*) is the minimum distance and *d* is designed to distance.

### 2.8. Galois Field

A finite field is called Galois field. Galois field extension of the polynomial ring *ℤ*_p_[*x*] is

(8) $$\begin{array}{c} \text{GF}\left(p^{m}\right)=\frac{Z_{p}\left[x\right]}{\langle P\left(x\right)\rangle }, \end{array}$$

where *p* is prime and *P*(*x*) is a primitive, irreducible polynomial of degree *m* over *ℤ*_p_. Therefore,

(9) $$\begin{array}{c} \text{GF}\left(p^{m}\right)=\left\{a_{0}+\cdots +a_{m-1}x^{m-1}:a_{i}\in {\mathbb{Z}}_{p^{j}},\;\forall i=0,\;1,\ldots m-1\right\}. \end{array}$$

### 2.9. MDS (Maximum Distance Separable) Matrices

MDS (Maximum Distance Separable) matrices have many applications in data security and channel coding. They create diffusion in block cipher data. These matrices are constructed by using the elements of a finite field. MDS matrices are invertible because the inverse of the MDS matrix is used for the decryption of data. Nowadays, Reed Solomon codes and BCH codes construct MDS matrices.

### 2.10. Proposition

If *l* × *l* MDS matrices can be generated from BCH code [*n*, *k*, *d*] over Galois field GF(2^*m*^) then *m*, *l*, and *d* must satisfy

(10) $$\begin{array}{c} m\geq \log_{2}2l+1,\\ l+1\leq d\leq 2^{m}-l. \end{array}$$

### 2.11. Proposition

Let *g*(*x*) be the generator polynomial of [*n*, *k*] cyclic code over the field ℱ. Let *H* be the *k* × *n* − *k* matrix whose *j*th row is rem_*g*(*x*)_(*x*^*n*−*k*+*j*−1^) , *j*=1,2,3 …, *k*. Then, the canonical parity check and generator matrices of the code are

(11) $$\begin{array}{c} H=\left[A^{t}:I_{n-k}\right],\\ G=\left[I_{k}:-A\right]. \end{array}$$

### 2.12. Example

Suppose that *p*(*x*)=*x*^7^+*x*+1 is a primitive, irreducible polynomial of degree 8 and *α* is the primitive root of *p*(*x*) over *ℤ*_2_[*x*]. Then the elements of Galois field GF(2^7^) are shown in Table 1.

We want to construct the BCH code of length 127 with designed distance *d*=60. Then find minimal polynomials corresponding to each *α*^*i*^ where *i*=1,2,3,   …, 59. By using Theorem 2.4. and elements of the Galois field from Table 1, we get the following distinct minimal polynomials.

Now, by taking the LCM of all minimal polynomials from Table 2, we get generator polynomial of degree 119 for 127 length BCH code.

(12) $$\begin{array}{c} g\left(x\right)=X^{119}+\;X^{117}+\;X^{115}+\;X^{113}+\;X^{112}+\;X^{109}+\;X^{108}+\;X^{104}+\;X^{100}+\;X^{98}\\ +\;X^{97}+\;X^{95}+\;X^{92}+\;X^{91}+\;X^{90}+\;X^{87}+\;X^{82}+\;X^{79}+\;X^{77}+\;X^{74}+\;X^{71}+\;X^{70}\\ +\;X^{68}+\;X^{67}+\;X^{65}+\;X^{64}+\;X^{63}+\;X^{59}+\;X^{58}+\;X^{57}+\;X^{56}+\;X^{54}+\;X^{48}+\;X^{47}\\ +\;X^{45}+\;X^{43}+\;X^{39}+\;X^{38}+\;X^{35}+\;X^{33}+\;X^{32}+\;X^{31}+\;X^{29}+\;X^{28}+\;X^{23}+\;X^{22}\\ +\;X^{21}+\;X^{19}+\;X^{17}+\;X^{16}+\;X^{15}+\;X^{14}+\;X^{11}+\;X^{10}+\;X^{9}+\;X^{8}+\;X^{7}+\;X^{5}+\;X^{4}\\ +\;X^{3}+\;X^{2}+\;X+1. \end{array}$$

## 3. Proposed Algorithm

In this algorithm, the key and block size are 128 bits. Simple logical and arithmetic operations are like shifting and logical XOR. Mainly, 2 steps are repeated 10 times for encrypting plain image data. These two steps are not constant for each round. Perhaps these steps introduced new entry in the next round, making the cryptanalysis more difficult.

### 3.1. Steps of Encryption

- Step 1: convert 128 bits of data into 16 data bytes and write these 16 bytes into a 4*∗*4 state matrix.
- Step 2: construct keys using the BCH codes of length 128 by taking different designed distances over the Galois field, used as round keys. Key 0 is used in round 0; key 1 is used in round 1. Apply all 10 different keys in 10 rounds.
- Step 3: ten different MDS matrices are constructed for each round using the BCH codes over the Galois field. Then the current state matrix is multiplied with the different MDS matrix in each round. The multiplication is modulo multiplication over the Galois field GF(2^8^).
- Step 4: then, take the analyses of the encrypted image and compare it with the original image.

### 3.2. Construction of Round Keys

The construction technique of round keys is followed by the binary representation of the generator polynomials of BCH codes over GF(2^7^) for different designed distances. Convert each generator polynomial to its binary representation form of length 128 bits. If it is not 128 bits, add check bits on the left-hand side to make 128 bits long. Then convert the BCH of length 128 into 16 bytes. This 16-byte string serves as a round key. Key 1 is derived from the generator polynomial of BCH code [*n*=127, *k*=1] with designed distance 65. By using the proposed technique, we get Key 1 as follows:

(i) Key 1: 127 255 255 255 255 255 255 255 255 255 255 255 255 255 255 255
  - Now we construct the next key by using BCH code of length 127 over Galois field GF(2^7^) with a designed distance of 60. Then convert the coefficients of generator polynomial *g*(*x*) which are in descending order into the block of 8 bits.
  - 00000000 10101011 00110001 00010110 10011100 10000100 10100100 11011011 10001111 01000001 10101000 11001011 10110000 11101011 11001111 10111111
  - Convert each byte into the decimal form so that key 2 is as follows:
(ii) Key 2: 0 171 49 22 156 132 164 219 143 65 168 203 176 235 207 191
  - Similarly, we construct all keys using BCH codes over the Galois field by changing the designed distance.
(iii) Key 3: 0 1 101 123 192 163 7 249 56 40 16 229 154 109 22 187
(iv) Key 4: 0 0 3 146 27 208 157 120 3 122 83 250 137 174 174 43
(v) Key 5: 0 0 0 5 16 109 174 23 166 30 82 12 96 106 78 41
(vi) Key 6: 0 0 0 0 13 83 6 214 191 219 200 87 71 25 231 13
(vii) Key 7: 0 0 0 0 0 25 161 99 10 46 46 13 22 111 12 93
(viii) Key 8: 0 0 0 0 0 0 41 19 31 9 172 122 28 6 238 111
(ix) Key 9: 0 0 0 0 0 0 0 65 218 145 157 158 251 54 166 153
(x) Key 10: 0 0 0 0 0 0 0 0 244 132 85 24 185 88 42 31

### 3.3. Construction of Mixed Column Matrix

This is a significant step in the proposed algorithm which creates confusion and diffusion. We construct a mixed column matrix by following steps:

- Step 1: construct a generator polynomial of BCH code of length *n* with designed distance *δ* where *n*=2^*m*^ − 1 and *m* is the degree of the primitive, irreducible polynomial.
- Step 2: select a value *δ* satisfying *l*+1 ≤ *δ* ≤ 2^*m*^ − *l*.
- Step 3: calculate the dimension of the code, *k*=*n* − *r*, where *r* is the degree of the generator polynomial of BCH code.
- Step 4: divide the *x*^*n*−*k*+*i*−1^ where *i*=1,2,…*k* by generator polynomial and get remainder polynomial.
- Step 5: convert each remainder polynomial into binary form, make a block of 8 bits, and convert each block into decimal form.
- Step 6: write coefficients of the remainder polynomial, which are in decimal form, into *l* × *l* matrix such that matrix is nonsingular.

### 3.4. Demonstration

Suppose that we want to construct the MDS matrices with the help of BCH code of length 255 with designed distance *δ*  = 119. Here we take *l*=4, so that *δ* satisfies the inequality 5 ≤ *δ* ≤ 252. Generator polynomial is for BCH code with [*n*=255, *k*=13, *δ*=119]. The coefficients of generator polynomial in descending form are as follows:

101101010011001110000010100010111111111001010111011111100101100110000100111111011011100000011101101011111101000110111000100001011101000010110011100100011000010000010010000100100101111001100001110100001100010001000100101001011111010100010010111.

We find the remg_*BCH*_(*x*)(*x*^*n*−*k*+*i*−1^),  *i*=1,…, 13, that is, remg_*BCH*_(*x*)(*x*^*i*+241^). Coefficients of the polynomial remg_*BCH*_(*x*)(*x*^242^) are into the block of 8 bits. Here remg_*BCH*_(*x*)(*x*^242^) is the remainder polynomial after dividing *x*^242^ by generator polynomial of BCH code. The coefficients of remainder polynomial are as follows.

11101001 00010101 11110100 10100100 01000100 01100001 01110000 11001111 01001001 00001001 00000100 00110001 00111001 10100001 01110100 00100011 10110001 01111110 10110111 00000011 10110111 11100100 00110011 01001111 11011101 01001111 11111010 00101000 00111001 10010101 110100100

(13) $$\begin{array}{c} A=\left[\begin{array}{cccc} 11101001 & 01000100 & 01001001\; & 00111001\\ 00010101 & 01100001 & 00001001 & 10100001\\ 11110100 & 01110000 & 00000100 & 01110100\\ 10100100 & 11001111 & 00110001 & 00100011 \end{array}\right]. \end{array}$$

Now, converting each block into decimal form

(14) $$\begin{array}{c} A=\left[\begin{array}{cccc} 233 & 68 & 73\; & 57\\ 21 & 97 & 9 & 161\\ 244 & 112 & 4 & 116\\ 164 & 207 & 49 & 35 \end{array}\right]. \end{array}$$

Similarly, we construct 9 more MDS matrices for each round using BCH codes of length 127 corresponding to different designed distances for the image encryption scheme.

(15) $$\begin{array}{c} A_{1}=\left[\begin{array}{cccc} 221 & 104 & 182\; & 89\\ 110 & 180 & 91 & 44\\ 234 & 50 & 155 & 207\\ 168 & 113 & 251 & 190 \end{array}\right],\\ A_{2}=\left[\begin{array}{cccc} 212 & 117 & 117\; & 145\\ 190 & 79 & 207 & 89\\ 95 & 39 & 231 & 172\\ 251 & 230 & 134 & 71 \end{array}\right],\\ A_{3}\left[\begin{array}{cccc} 148 & 114 & 86\; & 6\\ 74 & 57 & 43 & 3\\ 177 & 110 & 195 & 135\\ 88 & 183 & 87 & 195 \end{array}\right],\\ A_{4}=\left[\begin{array}{cccc} 176 & 231 & 152\; & 226\\ 232 & 148 & 84 & 147\\ 196 & 173 & 178 & 171\\ 98 & 86 & 217 & 85 \end{array}\right],\\ A_{5}=\left[\begin{array}{cccc} 186 & 48 & 246\; & 104\\ 231 & 40 & 141 & 92\\ 201 & 164 & 11 & 198\\ 222 & 226 & 174 & 11 \end{array}\right],\\ A_{6}=\left[\begin{array}{cccc} 246 & 119 & 96\; & 56\\ 123 & 59 & 176 & 28\\ 203 & 234 & 184 & 54\\ 101 & 245 & 92 & 27 \end{array}\right],\\ A_{7}=\left[\begin{array}{cccc} 153 & 101 & 108\; & 223\\ 76 & 178 & 182 & 111\\ 38 & 89 & 91 & 55\\ 19 & 45 & 173 & 155 \end{array}\right],\\ A_{8}=\left[\begin{array}{cccc} 248 & 84 & 26\; & 157\\ 132 & 126 & 23 & 83\\ 66 & 63 & 11 & 233\\ 33 & 31 & 133 & 244 \end{array}\right],\\ A_{9}=\left[\begin{array}{cccc} 136 & 52 & 201\; & 200\\ 68 & 26 & 100 & 228\\ 34 & 13 & 50 & 114\\ 153 & 50 & 80 & 241 \end{array}\right]. \end{array}$$

These are the required matrices used in the proposed algorithm in the mixed column transformation step for image data security.

## 4. Analysis

### 4.1. Key Space Analysis

The asset of an algorithm of cryptography depends on the space of the key, so the length of the key must be large for a brute force attack. The proposed algorithm has 2^128^ possible keys, which are very large. Suppose any unauthorized person tries for a brute force attack. In that case, the acute sensitivity is very high for this algorithm, so he has to try all possibilities of keys for the decryption of the image, which is very difficult to do computationally.

### 4.2. Key Sensitivity Analysis

High key sensitivity is vital for image security, which means that the encrypted image cannot be converted into a plain image correctly even if there is a small change between decryption or encryption keys. The proposed algorithm is tested for different keys with a minimal difference. This is the same as an avalanche effect in text encryption, where a minimal change in the key gives a major difference in the encrypted text. The strength of an algorithm is that if a key is changed by a single bit, then the original image cannot be obtained.

### 4.3. Statistical Analysis for Image Encryption

Statistical analyses are used to determine the statistical features of the encryption technique. These analyses include correlation, information entropy, contrast, homogeneity, and energy. These analyses determine the strength of the encryption scheme. Statistical analyses decide whether the encryption scheme is secure for image encryption or not. The details of statistical analyses are briefly discussed as follows.

#### 4.3.1. Histogram Analysis

Histogram analysis is used to see how much encryption procedure is needed to change test image compared to the encrypted image. For good encryption, the histogram of the ciphered image should have a uniform distribution that indicates that the anticipated scheme can resist statistical attacks.  Figure 1–6 shows the histogram analysis of test images and encrypted images.  Figure 1 shows original image histogram and Figure 4 shows the histogram of encrypted image through blue channel.  Figure 2 shows histogram of original image and Figure 5 shows histogram of encrypted image through green channel.  Figure 3 is showing histogram of plain image and Figure 6 shows histogram of encrypted image through red channel.

The histograms of the ciphered images are appreciably uniform and are quite dissimilar from the test images. The suggested encryption technique has fulfilled all the test image features and has convoluted the statistical bond between the test image and its cipher image.

#### 4.3.2. Contrast

Contrast analysis organizes the objects in an image. A secure encryption technique has high contrast values. It measures the color difference, which identifies the distinctive in an object. More briefly, it measures the change in brightness, color, and other objects within a similar frame of view. Contrast can be measured mathematically by the equation

(16) $$\begin{array}{c} C=\underset{g,h}{\sum }{\left|g-h\right|}^{2}n\left(g,h\right). \end{array}$$

*n*(*g*, *h*) denotes the number of grey-level cooccurrence matrices and *g*, *m* are the pixels of an image. The strength of contrast between the pixels and their adjacent pixels is compared in the full image.

#### 4.3.3. Correlation

The correlation analysis is used to break the relationship between the neighboring pixels. The test image correlation is approaching one. The encrypted image should correlate coming zero for better encryption. To determine the encryption effect of the proposed technique, perform correlation analysis on the plain and encrypted image. The correlation coefficient is calculated by formula

(17) $$\begin{array}{c} r_{xy}=\frac{E\left(\left(x-{µ}_{x}\right)\left(y-{µ}_{y}\right)\right)}{\sqrt{\delta x\delta y}}. \end{array}$$

*δ* and *µ* and denote the variance and expected value.

#### 4.3.4. Energy

In this analysis, we compute the energy of the encrypted images by applying S-boxes. This measure gives the sum of squared elements in the grey-level cooccurrence matrix

(18) $$\begin{array}{c} e=\sum_{l,m}p{\left(l,m\right)}^{2}, \end{array}$$

where *p*(*l*, *m*) is the number of grey-level cooccurrence matrices.

#### 4.3.5. Homogeneity

In homogeneity, the grey-level cooccurrence matrix explains the proficiency of arrangements of pixel brightness results in tabular form. The closeness of the distribution in the grey-level cooccurrence matrix to its diagonal is measured through the homogeneity analysis. If the homogeneity is as small as possible, then encryption is better. The following formula measures homogeneity:

(19) $$\begin{array}{c} H=\sum_{l,m}\frac{n\left(l,m\right)}{1+\left|l-m\right|}. \end{array}$$

#### 4.3.6. Entropy

Information entropy measures the disorder which is created by the encryption process. Entropy measures the strength of the encryption technique. An encryption technique is good if it has more disorder and randomness. Entropy is defined as

(20) $$\begin{array}{c} e=-\sum_{i=1}^{n}p\left(x_{i}\right)\log_{b}p\left(x_{i}\right), \end{array}$$

where *P*(*x*_*i*_) contains the histogram counts. Entropy must be close to 8 for better image quality.

#### 4.3.7. Image Encryption

The image is encrypted using the proposed scheme.  Figure 7 shows the original Lena image, and Figure 8 shows the encrypted Lena image. The comparison results of the original AES algorithm and proposed encryption technique are shown in Table 3.

Table 3 shows results of the encryption technique using the original AES algorithm and proposed AES algorithm through the red, green, and blue channels. The contrast of the proposed AES is better than the original AES. Correlation and energy are also close to zero. Proposed homogeneity is also good as compared to the original AES. Entropy is close to 8, which shows that our image encryption technique is good.

## 5. Conclusion

This paper encrypts the image using the novel technique based on BCH codes over the Galois field. We introduce a new method for image encryption using Bose Chaudhary Hocquenghem codes which secures our data. We constructed the secret keys and MDS matrices using the BCH codes of length 127 over the Galois field (2^7^). Then encrypt the image using the proposed modified AES algorithm. Table 3 concludes that the proposed image encryption technique is better than the original AES algorithm. Correlation, homogeneity, and energy of encrypted image also show promising results for image data security. Our histogram analysis shows that the proposed encryption scheme is improved. We can conclude that the proposed algorithm gives a high-security level to image data using different tests and studies. The unauthorized user cannot access the data without permission. This algorithm can be used in various intelligence agencies, Forensics, and Military Communication in the future. Further, this work can be extended to apply text, audio, video encryption.

## Figures and Tables

**Figure 1:** Original blue.

**Figure 2:** Original green.

**Figure 3:** Original red.

**Figure 4:** Encrypted blue.

**Figure 5:** Encrypted green.

**Figure 6:** Encrypted red.

**Figure 7:** Original image.

**Figure 8:** Encrypted image.

**Table 1:** Elements of Galois field GF(2^7^).

*α*	*α*^2	*α*^3	*α*^4
*α*^5	*α*^6	*α*^7 = *α* + 1	*α*^8 = *α*^2^ + *α*
*α*^9 = *α*^3^ + *α*^2^	*α*^10 = *α*^4^ + *α*^3^	*α*^11 = *α*^5^ + *α*^4^	*α*^12 = *α*^6^ + *α*^5^
*α*^13 = *α*^6^ + *α* + 1	*α*^14 = *α*^2^ + 1	*α*^15 = *α*^3^ + *α*	*α*^16 = *α*^4^ + *α*^2^
*α*^17 = *α*^5^ + *α*^3^	*α*^18 = *α*^6^ + *α*^4^	*α*^19 = *α*^5^ + *α* + 1	*α*^20 = *α*^6^ + *α*^2^ + *α*
*α*^21 = *α*^3^ + *α*^2^ + *α* + 1	*α*^22 = *α*^4^ + *α*^3^ + *α*^2^ + *α*	*α*^23 = *α*^5^ + *α*^4^ + *α*^3^ + *α*^2^	*α*^24 = *α*^6^ + *α*^5^ + *α*^4^ + *α*3
*α*^25 = *α*^6^ + *α*^5^ + *α*^4^ + *α* + 1	*α*^26 = *α*^6^ + *α*^5^ + *α*^2^ + 1	*α*^27 = *α*^6^ + *α*^3^ + 1	*α*^28 = *α*^4^ + 1
*α*^29 = *α*^5^ + *α*	*α*^30 = *α*^6^ + *α*^2^	*α*^31 = *α*^3^ + *α* + 1	*α*^32 = *α*^4^ + *α*^2^ + *α*
*α*^33 = *α*^5^ + *α*^3^ + *α*^2^	*α*^34 = *α*^6^ + *α*^4^ + *α*^3^	*α*^35 = *α*^5^ + *α*^4^ + *α* + 1	*α*^36 = *α*^6^ + *α*^5^ + *α*^2^ + *α*
*α*^37 = *α*^6^ + *α*^3^ + *α*^2^ + *α* + 1	*α*^38 = *α*^4^ + *α*^3^ + *α*^2^ + 1	*α*^39 = *α*^5^ + *α*^4^ + *α*^3^ + *α*	*α*^40 = *α*^6^ + *α*^5^ + *α*^4^ + *α*^2^
*α*^41 = *α*^6^ + *α*^5^ + *α*^3^ + *α* + 1	*α*^42 = *α*^6^ + *α*^4^ + *α*^2^ + 1	*α*^43 = *α*^5^ + *α*^3^ + 1	*α*^44 = *α*^6^ + *α*^4^ + *α*
*α*^45 = *α*^5^ + *α*^2^ + *α* + 1	*α*^46 = *α*^6^ + *α*^3^ + *α*^2^ + *α*	*α*^47 = *α*^4^ + *α*^3^ + *α*^2^ + *α* + 1	*α*^48 = *α*^5^ + *α*^4^ + *α*^3^ + *α*^2^ + *α*
*α*^49 = *α*^6^ + *α*^5^ + *α*^4^ + *α*^3^ + *α*^2^	*α*^50 = *α*^6^ + *α*^5^ + *α*^4^ + *α*^3^ + *α* + 1	*α*^51 = *α*^6^ + *α*^5^ + *α*^4^ + *α*^2^ + 1	*α*^52 = *α*^6^ + *α*^5^ + *α*^3^ + 1
*α*^53 = *α*^6^ + *α*^4^ + 1	*α*^54 = *α*^5^ + 1	*α*^55 = *α*^6^ + *α*	*α*^56 = *α*^2^ + *α* + 1
*α*^57 = *α*^3^ + *α*^2^ + *α*	*α*^58 = *α*^4^ + *α*^3^ + *α*^2^	*α*^59 = *α*^5^ + *α*^4^ + *α*^3^	*α*^60 = *α*^6^ + *α*^5^ + *α*4
*α*^61 = *α*^6^ + *α*^5^ + *α* + 1	*α*^62 = *α*^6^ + *α*^2^ + 1	*α*^63 = *α*^3^ + 1	*α*^64 = *α*^4^ + *α*
*α*^65 = *α*^5^ + *α*^2^	*α*^66 = *α*^6^ + *α*^3^	*α*^67 = *α*^4^ + *α* + 1	*α*^68 = *α*^5^ + *α*^2^ + *α*
*α*^69 = *α*^6^ + *α*^3^ + *α*^2^	*α*^70 = *α*^4^ + *α*^3^ + *α* + 1	*α*^71 = *α*^5^ + *α*^4^ + *α*^2^ + *α*	*α*^72 = *α*^6^ + *α*^5^ + *α*^3^ + *α*^2^
*α*^73 = *α*^6^ + *α*^4^ + *α*^3^ + *α* + 1	*α*^74 = *α*^5^ + *α*^4^ + *α*^2^ + 1	*α*^75 = *α*^6^ + *α*^5^ + *α*^3^ + *α*	*α*^76 = *α*^6^ + *α*^4^ + *α*^2^ + *α* + 1
*α*^77 = *α*^5^ + *α*^3^ + *α*^2^ + 1	*α*^78 = *α*^6^ + *α*^4^ + *α*^3^ + *α*	*α*^79 = *α*^5^ + *α*^4^ + *α*^2^ + *α* + 1	*α*^80 = *α*^6^ + *α*^5^ + *α*^3^ + *α*^2^ + *α*
*α*^81 = *α*^6^ + *α*^4^ + *α*^3^ + *α*^2^ + *α* + 1	*α*^82 = *α*^5^ + *α*^4^ + *α*^3^ + *α*^2^ + 1	*α*^83 = *α*^6^ + *α*^5^ + *α*^4^ + *α*^3^ + *α*	*α*^84 = *α*^6^ + *α*^5^ + *α*^4^ + *α*^2^ + *α* + 1
*α*^85 = *α*^6^ + *α*^5^ + *α*^3^ + *α*^2^ + 1	*α*^86 = *α*^6^ + *α*^4^ + *α*^3^ + 1	*α*^87 = *α*^5^ + *α*^4^ + 1	*α*^88 = *α*^6^ + *α*^5^ + *α*
*α*^89 = *α*^6^ + *α*^2^ + *α* + 1	*α*^90 = *α*^3^ + *α*^2^ + 1	*α*^91 = *α*^4^ + *α*^3^ + *α*	*α*^92 = *α*^5^ + *α*^4^ + *α*^2^
*α*^93 = *α*^6^ + *α*^5^ + *α*^3^	*α*^94 = *α*^6^ + *α*^4^ + *α* + 1	*α*^95 = *α*^5^ + *α*^2^ + 1	*α*^96 = *α*^6^ + *α*^3^ + *α*
*α*^97 = *α*^4^ + *α*^2^ + *α* + 1	*α*^98 = *α*^5^ + *α*^3^ + *α*^2^ + *α*	*α*^99 = *α*^6^ + *α*^4^ + *α*^3^ + *α*^2^	*α*^100 = *α*^5^ + *α*^4^ + *α*^3^ + *α* + 1
*α*^101 = *α*^6^ + *α*^5^ + *α*^4^ + *α*^2^ + *α*	*α*^102 = *α*^6^ + *α*^5^ + *α*^3^ + *α*^2^ + *α* + 1	*α*^103 = *α*^6^ + *α*^4^ + *α*^3^ + *α*^2^ + 1	*α*^104 = *α*^5^ + *α*^4^ + *α*^3^ + 1
*α*^105 = *α*^6^ + *α*^5^ + *α*^4^ + *α*	*α*^106 = *α*^6^ + *α*^5^ + *α*^2^ + *α* + 1	*α*^107 = *α*^6^ + *α*^3^ + *α*^2^ + 1	*α*^108 = *α*^4^ + *α*^3^ + 1
*α*^109 = *α*^5^ + *α*^4^ + *α*	*α*^110 = *α*^6^ + *α*^5^ + *α*^2^	*α*^111 = *α*^6^ + *α*^3^ + *α* + 1	*α*^112 = *α*^4^ + *α*^2^ + 1
*α*^113 = *α*^5^ + *α*^3^ + *α*	*α*^114 = *α*^6^ + *α*^4^ + *α*^2^	*α*^115 = *α*^5^ + *α*^3^ + *α* + 1	*α*^116 = *α*^6^ + *α*^4^ + *α*^2^ + *α*
*α*^117 = *α*^5^ + *α*^3^ + *α*^2^ + *α* + 1	*α*^118 = *α*^6^ + *α*^4^ + *α*^3^ + *α*^2^ + *α*	*α*^119 = *α*^5^ + *α*^4^ + *α*^3^ + *α*^2^ + *α* + 1	*α*^120 = *α*^6^ + *α*^5^ + *α*^4^ + *α*^3^ + *α*^2^ + *α*
*α*^121 = *α*^6^ + *α*^5^ + *α*^4^ + *α*^3^ + *α*^2^ + *α* + 1	*α*^122 = *α*^6^ + *α*^5^ + *α*^4^ + *α*^3^ + *α*^2^ + 1	*α*^123 = *α*^6^ + *α*^5^ + *α*^4^ + *α*^3^ + 1	*α*^124 = *α*^6^ + *α*^5^ + *α*^4^ + 1
*α*^125 = *α*^6^ + *α*^5^ + 1	*α*^126 = *α*^6^ + 1	*α*^127 = 1	0

**Table 2:** Minimal polynomials.

*M* (1) = *x*^7^ + *x* + 1
*M* (2) = *x*^7^ + *x*^5^ + *x*^3^ + *x* + 1
*M* (3) = *x*^7^ + *x*^3^ + *x*^2^ + *x* + 1
*M* (4) = *x*^7^ + *x*^6^ + *x*^5^ + *x*^4^ + *x*^3^ + *x*^2^ + 1
*M* (5) = *x*^7^ + *x*^5^ + *x*^4^ + *x*^3^ + 1
*M* (6) = *x*^7^ + *x*^3^ + 1
*M* (7) = *x*^7^ + *x*^6^ + *x*^5^ + *x*^2^ + 1
*M* (8) = *x*^7^ + *x*^5^ + *x*^4^ + *x*^3^ + *x*^2^ + *x* + 1
*M* (9) = *x*^7^ + *x*^6^ + *x*^5^ + *x*^3^ + *x*^2^ + *x* + 1
*M* (10) = *x*^7^ + *x*^6^ + *x*^3^ + *x* + 1
*M* (11) = *x*^7^ + *x*^5^ + *x*^2^ + *x* + 1
*M* (12) = *x*^7^ + *x*^6^ + *x*^5^ + *x*^4^ + *x*^2^ + *x* + 1
*M* (13) = *x*^7^ + *x*^4^ + 1
*M* (14) = *x*^7^ + *x*^6^ + *x*^4^ + *x*^2^ + 1
*M* (15) = *x*^7^ + *x*^6^ + *x*^4^ + *x* + 1
*M* (16) = *x*^7^ + *x*^6^ + *x*^5^ + *x*^4^ + 1
*M* (17) = *x*^7^ + *x*^4^ + *x*^3^ + *x*^2^ + 1

**Table 3:** Analyses of original and encrypted image

Channel	Contrast	Correlation	Energy	Homogeneity	Entropy
Original AES red	5.1454	0.0742	0.0254	0.4701	7.7337
Proposed AES red	5.2462	0.0731	0.0256	0.4661	7.7959
Original AES green	5.3501	0.0804	0.0250	0.4621	7.7337
Proposed AES green	5.3557	0.0800	0.0250	0.4620	7.7959
Original AES blue	5.0947	0.0721	0.0270	0.4666	7.7337
Proposed AES blue	5.1995	0.0716	0.0271	0.4602	7.7959

## Data Availability

No such type of data were used in this manuscript.
